The article "Analysis of Prescription Medication Rules of Traditional Chinese Medicine for Diabetes Treatment Based on Data Mining" was retracted in 2023. Reasons: signs of a paper mill; suspected computer-generated content; unreliable results or conclusions; concerns about the data.

# Analysis of Prescription Medication Rules of Traditional Chinese Medicine for Diabetes Treatment Based on Data Mining

**DOI:** 10.1155/2022/7653765

**Published:** 2022-01-31

**Authors:** Yi Zhang, Jun Hou, Ziyu Zeng

**Affiliations:** ^1^Preventive Health Department, Shanghai Municipal Hospital of Traditional Chinese Medicine, Shanghai University of Traditional Chinese Medicine, Shanghai 200071, China; ^2^Preventive Health Department, Shanghai Guangzhong Street Community Health Service Center, Shanghai 201203, China

## Abstract

In this study, we have used TCM medical record management platform and SAS statistical software to analyze the cases of a professor in the treatment of type 2 diabetes, in order to explore the medication rules for the treatment of type 2 diabetes, so as to enrich and optimize the diagnosis and treatment plan for type 2 diabetes based on the experience of famous doctors. Chinese medicine treatment provides more diagnosis and treatment ideas. We have collected the professor's treatment of type 2 diabetes, screened out 100 patients, from a total of 285 prescriptions, and entered them into the TCM medical record management platform. We used the TCM medical record management platform and SAS statistical software to analyze his professor's experience in the treatment of type 2 diabetes. The medication analysis is as follows: (1) frequency of medication: 285 cases that met the inclusion criteria used a total of 187 traditional Chinese medicines. Among them, Salvia miltiorrhiza was used most frequently; (2) drug frequency analysis: 285 cases met the inclusion criteria, and the four Qi were mainly cold and warm medicines. The five flavors are mainly sweet, bitter, and pungent drugs. The main meridians are the liver, spleen, and kidney; (3) drug efficacy and classification analysis: 285 cases met the inclusion criteria, and 285 cases met the inclusion criteria and the Chinese medicines involved are the most common medicines used for tonic, heat clearing, blood circulation, and stasis; (4) clustering of medications: 35 Chinese medicines with medication frequency ≥20% are divided into 11 categories. (5) Using the improved Apriori algorithm, the minimum confidence level is selected to be 0.5, data mining is conducted on all type 2 diabetes cases, and a total of 21 recipes are dug out involving 10 Chinese medicines. In this study, with the aid of the TCM medical record management platform and SAS statistical software, cluster analysis, improved Apriori algorithm, and other data mining methods were used to systematically and objectively analyze the professor's treatment of type 2 diabetes cases. The results have clinical significance and can be used for traditional Chinese medicine treatment of type 2 diabetes, which provides an objective basis and provides a certain reference for the current inheritance of traditional Chinese medical experience and summary research.

## 1. Introduction

Diabetes is a metabolic disease characterized by chronic hyperglycemia caused by a variety of causes and is caused by defects in insulin secretion and/or function [1]. DM is a common and frequently occurring disease, mainly type 1 diabetes and type 2 diabetes, among which T2DM is a common clinical type. In 2013, according to the International Diabetes Federation (IDF) statistics: at present, 382 million people worldwide are threatened by DM. It is estimated that in the next 25 years, the number of people suffering from DM will reach or exceed 592 million [2]. Today, about 80% of DM patients in the world live in middle- or low-income countries. The number of DM cases in my country is significantly higher than that in other countries, ranking first in the world. The prevalence of DM in my country is obviously more severe than that in other Western countries. At present, more than 90.0% of the people with DM in my country belong to T2DM, and only about 5.0% of the population belong to T1DM. Therefore, the majority of T2DM populations are in my country [3]. DM has become a public health issue of increasing concern worldwide. In many countries, DM and its various complications have become an important cause of disability, death, and increased medical expenses. Therefore, the prevention and treatment of DM cannot be delayed. At present, the treatment of T2DM in Western medicine mainly includes oral hypoglycemic drugs and insulin for injection. Although it can stabilize blood sugar, there are still many problems in relieving patients' clinical symptoms and treating various complications.

The name “diabetes” does not appear in ancient Chinese classics. According to the typical clinical manifestations of this disease, T2DM is generally classified as “diabetes.” Traditional Chinese medicine has a long history of prevention and treatment of diabetes. From the record of “Diabetes” in the “Huang Di Nei Jing,” with the continuous accumulation of clinical experience, TCM has deepened the understanding of diabetes. Traditional Chinese medicine has obvious advantages in alleviating various clinical symptoms of DM, preventing and treating various complications, and improving the quality of life of DM patients. Based on this, this study collected the cases of treatment of T2DM and used a variety of data mining methods with the aid of the medical record management platform and SAS statistical software to analyze the law of the treatment of T2DM as shown in Figure 1 and provide a basis for the treatment of T2DM in T2DM, thereby strengthening that Chinese medicine intervention for T2DM can relieve the clinical symptoms of T2DM patients and improve the quality of life.

Data mining is translated into data mining and data exploration and is usually related to computer science. Data mining is one of the disciplines that has gradually emerged to solve the problem of “rich data but poor knowledge.” It generally refers to extracting a large number of random, fuzzy, and incomplete data from large databases through various algorithms that are not understood by people, are inherently hidden, but have practical value to people and effective potential information and knowledge. In a nutshell, data mining refers to the process of discovering or extracting valuable information from a large amount of chaotic data [4]. The main function of data mining is prediction and description. In simple terms, the process can be divided into three stages: firstly, the required data are obtained through various methods, and then, the data are normalized [5]; secondly, the law of connection between data and data through various channels is sought; and finally, the acquired laws are presented completely in a way that can be understood by users [6]. At present, the specific implementation of data mining has also become rich and diverse, mainly including information retrieval, machine learning, statistical analysis, and pattern recognition, enabling data mining technology to be used in various fields around the world such as basic medicine, epidemiological research, disease diagnosis and treatment, medical statistical methodology, genetics, and other aspects, which have been widely used [7–10] and have achieved remarkable results.

This research uses a variety of data mining methods to systematically analyze an in-depth excavation of a professor's clinical treatment of T2DM cases with the help of the Chinese medical record management platform and SAS statistical software, mainly from the frequency of medication, drug frequency analysis, the efficacy and classification of medication, and medication clustering, and improved Apriori algorithm and other aspects are carried out, to inherit and carry forward the academic thought and clinical experience of the tutor in the clinical treatment of T2DM and provide more diagnosis and treatment ideas for T2DM treatment, which has important practical significance and clinical value.

In this study, we have used TCM medical record management platform and SAS statistical software to analyze the cases of a professor in the treatment of type 2 diabetes, in order to explore the medication rules for the treatment of type 2 diabetes, so as to enrich and optimize the diagnosis and treatment plan for type 2 diabetes based on the experience of famous doctors. Chinese medicine treatment provides more diagnosis and treatment ideas. We have collected the professor's treatment of type 2 diabetes, screened out 100 patients, from a total of 285 prescriptions, and entered them into the TCM medical record management platform. He used the TCM medical record management platform and SAS statistical software to analyze his professor's experience in the treatment of type 2 diabetes. The medication analysis is as follows:

1. Frequency of medication: 285 cases that met the inclusion criteria used a total of 187 traditional Chinese medicines. Among them, Salvia miltiorrhiza was used most frequently.
2. Drug frequency analysis: 285 cases met the inclusion criteria, and the four Qi were mainly cold and warm medicines. The five flavors are mainly sweet, bitter, and pungent drugs. The main meridians are the liver, spleen, and kidney.
3. Drug efficacy and classification analysis: 285 cases met the inclusion criteria, and the Chinese medicines involved are the most common medicines for tonic, blood circulation and blood stasis, and heat-clearing medicines.
4. Clustering of medications: 35 Chinese medicines with medication frequency ≥20% are divided into 11 categories.
5. Using the improved Apriori algorithm: the minimum confidence level is selected to be 0.5, data mining is conducted on all type 2 diabetes cases, and a total of 21 recipes involving 10 Chinese medicines are dug out.

The rest of this manuscript is arranged as follows.

In section 2, a brief summary of the related work, which is already available in the literature, is presented, which is followed by a detailed explanation of the proposed methodology and its effectiveness in resolving the aforementioned issues. In section 4, experimental results and observations are thoroughly analyzed from various perspectives. Finally, concluding remarks are given at the end along with references.

## 2. Related Work

Zu [11] believed that dryness and dampness have the same disease, phlegm and dampness are stagnant, and body fluid is not distributed. Dryness is easy to damage body fluid, body tract obstruction, and abnormal Qi, and dampness is caused by evil. Therefore, the theory of “dampness and dampness simultaneous treatment” should run through the whole process of diabetes, and the method of promoting body fluid and moisturizing dryness should be taken into consideration while strengthening the spleen and dispelling dampness. Li et al. [12] believed that heat is the initial cause of the disease and it runs through the whole process of T2DM. It is proposed to use the heat-clearing method to treat T2DM, and the heat-clearing drugs are divided into the following three categories: (i) severe cold such as coptis, scutellaria, phellodendron, and gypsum; (ii) medium cold such as tree peony, honeysuckle, red peony root, and prunella vulgaris; and (iii) continuous or ordinary such as light bamboo leaves and mulberry branches. He also pointed out that care should be taken to protect the spleen and stomach while clearing away heat. Adhering to the treatment principles of clearing away heat, detoxifying, and nourishing yin, purging fire and detoxification should consolidate the root cause. These have important reference value for clinical diagnosis and treatment of diabetes. Du [13] believed that turbid toxins run through diabetes, and the prevention and treatment of diabetes should focus on the application of clearing away heat and detoxification, resolving turbidity and detoxification, replenishing Qi, and nourishing and detoxifying Yin, to achieve good results. Zhu [14] creatively proposed the method of promoting blood circulation to remove blood stasis for the treatment of diabetes and its complications for the first time. At the same time, he paid attention to regulating the relationship between Qi and blood.

Feng [15] believed that “the spleen governs movement” is a prerequisite for “spleen control,” and the loss of spleen transformation is the key to the pathogenesis of diabetes. Diabetes is treated according to the perspective of spleen transformation and loss of division: spleen deficiency is not transformed, and this type is mostly a syndrome of deficiency and excess. The treatment should be based on the principle of “deficiency to replenish it, but to reduce it in reality”; hypersplenism type: in this type, mostly the spleen and stomach accumulate heat, eliminate hunger, and relieve hunger. The treatment should be based on the principle of “heat and cold,” and the addition and subtraction of Yunu Decoction are chosen. Professor Zhu [16] based on the viewpoint of “Yang governs Yin from” proposed that the main pathologies of diabetes are liver, spleen, and kidneys. The basic pathogenesis is the deficiency of Yang of the spleen and kidney and the unfavorable cardinal mechanism. The warming Yang method is emphasized as the basic treatment method for diabetes, and at the same time, the three sour products of Schisandra, White Peony, and Cornus are commonly used to converge the vacant Yang Qi in the body and converge the power of the medicine to warm the Yang. The compatibility of warming Yang and acid collection is in line with the basic pathogenesis of this disease. Wang [17] pointed out that the occurrence and development of this disease are closely related to the liver. The overall goal of clinical treatment should be to restore the liver's function of regulating the flow of excretion. The basic principles of treatment should be to regulate and soothe the liver and also to soften and nourish the liver. Bupleurum, Bergamot, Angelica, Chuanmeizi, and White Peony are often chosen. Often choose Bupleurum, Bergamot, Angelica, Chuanmeizi, and White Peony along with other medicines for soothing liver and regulating Qi. At the same time, it is emphasized that while regulating the liver and soothing the liver, we should pay attention to protecting the spleen and stomach. Gao [18] believed that the pathogenesis of diabetes is mainly kidney Yin deficiency and dryness and heat as the standard. In the treatment, it mainly focuses on nourishing Yin and tonifying kidney, replenishing Qi, and nourishing Yin, and according to the different complications, it also uses tonifying kidney and warming Yang and promoting blood circulation.

Chen [19] treated T2DM from the four types such as lung and stomach dry heat type, Qi and Yin deficiency type, Yin and Yang deficiency type, and kidney deficiency and blood stasis type. Wang [20] treated T2DM according to five types: kidney Yin deficiency, dry heat injures in the lung, stomach dryness and body fluid injury, Yin deficiency and Yang floating, and Yin and Yang deficiency. The total effective rate of the treatment group is 90.33%. Ma [21] treated T2DM from 5 types of deficiency of both Yin and Yang, deficiency of both Qi and Yin, deficiency of liver and kidney, excess of Yin and heat, and internal accumulation of damp heat. The total effective rate in the treatment group was 97.96%.

Liu [22] based on the main theoretical basis of “strengthening fire to eat Qi, and Qi to eat less fire” divided the pathogenesis of T2DM into the following three stages: the early stage of strong fire and internal burning of the disease, and the clinical manifestation is liver and stomach stagnation and heat. The treatment should adhere to the principle of “remove the heat and eliminate the heat,” with aachaihu decoction as the main prescription; strengthening the fire and Qi is the middle stage of the disease, and this period is mainly caused by the burning of the Yin Qi for a long time. The clinical manifestations of Yin deficiency and dryness and heat often occur. The main principle of treatment is to replenish Qi and nourish Yin and at the same time to clear away heat. The main prescription is Baihu plus ginseng decoction; Qi, eating, and Yin and Yang are mainly seen in this stage. In the treatment, the main treatment is to promote blood circulation, remove blood stasis, and dredge collaterals, and also to warm the kidney Yang, in order to slightly generate fire and reduce the fire to get angry. At this stage, the Jinkui Shenqi Pill is the representative prescription.

## 3. Proposed Methodology

### 3.1. Research Standard

#### 3.1.1. Diagnostic Criteria

With reference to the relevant chapters in the “Guiding Principles for Clinical Research of New Chinese Medicines” [23], the following diagnostic criteria for syndrome types are proposed to be set.

1. Qi and Yin deficiency syndrome: fatigue, fatigue, thirst, and dry throat
2. Yin deficiency and heat syndrome: dry throat, thirst, upset, and irritability
3. Damp heat and sleepy spleen syndrome: full abdominal distension, heavy head, and body sleepiness
4. Blood stasis and collaterals syndrome: pain in the chest, flanks, waist and back, or tingling, and numbness of the limbs.
5. Deficiency of Yin and Yang, blood stasis, and water stop syndrome: weakness of waist and knees, insomnia and dreaminess, fatigue, and weakness

#### 3.1.2. Inclusion Criteria

This article uses the following inclusion criteria:

1. Those who meet the above diagnostic criteria
2. There is no restriction on gender, 18–80 years old
3. The number of patient visits is at least 2 times
4. Those who have been systematically treated by a professor and have complete medical records
5. Those who take traditional Chinese medicine decoction regularly

#### 3.1.3. Exclusion Criteria

This article uses the following exclusion criteria:

1. Those who do not meet the above diagnostic criteria and inclusion criteria
2. Those who have incomplete case data due to various factors
3. Women who are pregnant or breastfeeding
4. Those who are diagnosed with type 1 diabetes and other types of diabetes
5. With patients with severe heart, liver, and kidney dysfunction or other serious diseases of various systems
6. Those who are allergic to the relevant drugs in the treatment plan
7. Those who have acute complications such as diabetic ketoacidosis or co-infection within the past six months

#### 3.1.4. Case Rejection and Dropout Criteria

This article uses the following case rejection and dropout criteria:

1. Those who have incomplete data and affect the result statistics
2. Those who have a diagnosis without a prescription or only have dietary prescriptions
3. Those who change prescriptions for the purpose of nontreatment of diabetes
4. Those who have not taken traditional Chinese medicine decoctions as prescribed
5. Those who have serious adverse reactions during treatment and are unwilling or unsuitable to continue receiving treatment
6. Those who are lost to follow-up or the patient does not come to the clinic for follow-up visits on time

### 3.2. Clinical Information

All the collected case data are obtained from a professor at the Affiliated Hospital of Shandong University of Traditional Chinese Medicine and the Second Affiliated Hospital of Shandong University of Traditional Chinese Medicine between March 2018 and December 2018. The outpatient treatment of endocrinology department met the inclusion criteria for type 2 diabetes patient. Among them, there were 55 males and there were 45 females, with a total of 100 patients, and a total of 285 prescriptions were screened.

### 3.3. Data Entry

The collected 285 valid cases of type 2 diabetes were input into the TCM medical record management platform as required, mainly including basic information such as the patient's name, age, and gender, as well as information on four diagnoses, (i) TCM and Western medicine diagnosis, (ii) TCM syndrome types, (iii) treatment methods prescriptions, and (iv) drug administration methods. After the entry is completed, two people are responsible for reviewing the data to ensure the accuracy of the entered data and provide guarantee for the accuracy of the results.

### 3.4. Research Method

#### 3.4.1. Basic Information

The TCM medical record management platform is entered, “Diagnosis Statistics” in the statistical analysis is clicked, and the query conditions are entered. This condition was diagnosed by Western medicine as type 2 diabetes and Chinese medicine as diabetes. Statistics by gender and statistics by age are selected in the statistical results, respectively, and then, the corresponding tables or graphs can be drawn in turn.

#### 3.4.2. Analysis of TCM Medical Record Management Platform

The TCM medical record management platform is opened, the “sequence of drug properties” is clicked in the knowledge acquisition, and the query conditions are entered. This condition was diagnosed by Western medicine as type 2 diabetes and Chinese medicine as diabetes. You can get the frequency, efficacy, and classification frequency of Chinese medicine used in all type 2 diabetes cases, and the corresponding table or chart is obtained.

#### 3.4.3. Drug Analysis Based on SAS Statistical Software

Cluster analysis of medication use: all type 2 diabetes cases are entered into the TCM medical record management platform, and the statistical conditions are entered. This condition is diagnosed by Western medicine as type 2 diabetes and TCM as diabetes, and then, export “SAS” is clicked to obtain the required data set. Then, the obtained data set is imported into SAS through the import data function in SAS statistical software named sasuser.xj. Finally, the VARCLUS clustering process was used to perform cluster analysis of 35 drugs with medication frequency ≥20% in all cases.

#### 3.4.4. Drug Analysis Based on Improved Apriori Algorithm

All 285 cases of type 2 diabetes are entered into the TCM medical record management platform for data mining, the “drug combination” is clicked in the knowledge acquisition, and the corresponding query conditions are entered. A minimum confidence of 0.5 is chosen, and then, data mining on all type 2 diabetes cases is conducted.

### 3.5. Statistical Processing

#### 3.5.1. Drug Cluster Analysis

Using the VARCLUS clustering process provided by SAS statistical software (version 9.1), cluster analysis was performed on 35 drugs with medication frequency ≥20% in all cases.

#### 3.5.2. Drug Analysis Based on Improved Apriori Algorithm

The steps of the Apriori algorithm for mining frequent sets are as follows: the database to find frequent itemset is scanned, then frequent itemset is found through frequent itemset, and it is repeated until no more items can be found. From item set *L*_(*k* − 1)_ to *L*_*k*_, two steps are used to connect and delete. (1) Connection step: in order to find item set *L*_*k*_, two items in *L*_(*k* − 1)_ are connected to obtain a candidate set *C*_*k*_. (2) Deletion step: candidate set *C*_*k*_ is a superset of item set *L*_*k*_ and, therefore all frequent sets are included in it. However, itemsets are not necessarily frequent sets and are smaller than the minimum support need to be deleted. Finally, *L*_*k*_ is obtained.

## 4. Experiments and Discussion

### 4.1. Basic Information

In this study, a total of 100 T2DM patients met the inclusion criteria, including 55 males and 45 females, with a male-to-female ratio of 1.2 : 1. See Figure 2 for details.

In this study, there were 100 T2DM patients who met the inclusion criteria, and those over 40 years old accounted for 84.9% of all patients. See Figure 3 for the specific age distribution.

Basically, no significant difference in gender was observed, but overall males are slightly higher than females.

Judging from the statistics of age groups, 60–70 years of age group has the highest number of cases. Before the age of 70, the prevalence rate gradually increases with age. The decrease in the number of patients over 70 years of age in this study may be related to the number of collected cases. In this study, patients over the age of 40 accounted for 84.9%. The patients were mostly middle-aged and elderly. The results of the study are consistent with Wu Bin's report. The results of the study remind us that we must strengthen the prevention and active treatment of T2DM in the middle-aged and elderly population as soon as possible and enhance the awareness of prevention.

### 4.2. Analysis of TCM Medical Record Management Platform

There were 285 T2DM cases that met the inclusion criteria, involving a total of 187 Chinese medicines. Cold and warm drugs are used most frequently as shown in Figure 4.

The four Qi analyses of traditional Chinese medicine showed that the Chinese medicine used in 285 T2DM cases that met the inclusion criteria was involved in cold, heat, warm, and normal, but cold medicine and warm medicine were the main ones, all of which were ≥30%. Cold can clear away heat, purify fire, nourish Yin, warm to dispel lumps, warm up, and divert water. The instructor believes that for the common syndrome types of T2DM, heat syndromes are more common in Yin deficiency such as dry heat, heat toxin, damp heat, and stasis heat and Yin deficiency leads to heat, so drugs such as Coptis, Danshen, and Shengdi are often used to clear heat, relieve fire, and nourish Yin. The cold syndrome is more common in Yang deficiency, drinking water, blood stasis, and so on. Drinking is Yin evil and getting Yang will transform it to useful. If the blood is cold, it will condense, and if it is warm, it will do. At the same time, drugs that are too cold may cause blood stasis to block the collaterals. Water drinking and blood stasis are more common in the later stages of T2DM, with edema, numbness of the limbs and joints, and pain as the main manifestations. Instructors often choose astragalus, lychee seeds, atractylodes, and other drugs with warm nature to dispel cold, relieve pain, diure water, and promote the normal transfusion of body fluid and the smooth flow of Qi and blood. It can be seen that in the clinical treatment of T2DM, the instructor pays attention to both attack and tonic, and the combination of heat-clearing and heat-warming tonic.

There were 285 T2DM cases that met the inclusion criteria, involving a total of 187 Chinese medicines. Among them, sweet, bitter, and pungent drugs are used most frequently, as shown in Figure 5.

Among the 285 T2DM cases that met the inclusion criteria, the three drugs of sweet, bitter, and pungent were used most frequently. This reflects that the instructor pays attention to the theory of medicinal properties in the clinical treatment of T2DM and adheres to the principle of replenishing Qi and nourishing Yin, supplemented by clearing heat, and at the same time, it also pays attention to regulating the relationship between Qi and blood as the principle of diagnosis and treatment.

### 4.3. Drug Analysis Using SAS Statistical Software

Cluster analysis of medication use: among 285 T2DM cases that met the inclusion criteria, Chinese medicines are classified: Class 10 contains only 1 Chinese medicine without second characteristic roots, and the remaining 10 classes contain 2–5 Chinese medicines with second characteristic roots, all are less than 1. In the table, R-squared with own cluster represents the square of the correlation coefficient between the variable and the class component of the class. R-squared with next closest represents the square of the correlation coefficient between the variable and another type of component with second correlation, 1 − *R*^2^ ratio = (1 − *R* − squared with own cluster)/(1-R-squared with next closest). See Table 1 for details. ROC is R-squared with own cluster. RNC is R-squared with next closest.

The R-squared with own cluster value and *R*-squared with next closest value of the first class of drugs are both small, and the 1 − *R*^2^ ratio value is too large. This group of drugs treats T2DM patients with Qi stagnation, blood stasis, and heat toxin. The second category is mostly used to treat patients with T2DM of Qi deficiency and blood heat type. Class 3 drugs are mostly used to treat patients with T2DM of Qi stagnation and blood stasis. In the fourth category, this group of drugs is used to treat kidney deficiency patients with weak waist and knees as the main manifestation. Class 5 drugs are mostly used for the treatment of Yin deficiency and heat and blood stasis. Class 6 drugs for the treatment of blood stasis are mainly manifested by pain in the chest, waist, and back, fixed pain, or numbness or tingling. Class 7 drugs are mostly used for those with deficiency of both Qi and Yin with fatigue, dry mouth, and thirst as the main manifestations. Class 8 drugs are mostly used to treat Yin deficiency and blood heat with dry mouth, upset, and fear of heat as the main manifestations. Class 9 drugs are mostly used to treat spleen Qi deficiency, Yin deficiency, and internal heat, mainly manifested by abdominal distension and general weakness. Class 10 and Class 11 drugs are mostly used to treat patients with kidney Yang deficiency and swelling of the limbs.

### 4.4. Drug Analysis Results Based on the Improved Apriori Algorithm

The improved Apriori algorithm is used to select the minimum confidence level of 0.5, and data mining is performed on all T2DM cases that met the inclusion criteria. As a result, a total of 10 prescriptions were excavated. The specific frequency is as shown in Figure 6.

A total of 21 drug combinations were unearthed for all T2DM cases that met the inclusion criteria. These 21 drug combinations have clinical significance. A total of 10 Chinese medicines are involved: Salvia, Scrophulariaceae, Cangzhu, Pueraria, Atractylodes, Coptis, *Astragalus*, Mulberry Branch, Ghost Arrow Feather, and Wolfberry. These 10 drugs are the core drug combination used by the instructor to treat T2DM and the basic prescription for the instructor in the clinical treatment of T2DM.

## 5. Conclusion

In this study, with the help of the medical record management platform of Ming Lao TCM network and SAS statistical software, a variety of data mining methods such as medication clustering and improved Apriori algorithm are used to conduct in-depth mining and systematic analysis of a professor's treatment of T2DM cases to make his academic thinking clinical experience has been inherited and developed, providing new diagnosis and treatment ideas and objective basis for T2DM treatment with traditional Chinese medicine. The results of the study found that (1) frequency of medication: 285 cases that met the inclusion criteria used a total of 187 Chinese medicines, among which Danshen was used most frequently. (2) Analysis of the frequency of drug properties: the four Qi are mainly cold and warm drugs. The five flavors are mainly sweet, bitter, and pungent drugs. Guijing is mainly composed of liver, spleen, and kidney meridians. (3) Efficacy and classification analysis of medications: the effects of traditional Chinese medicines involved are mostly Qi-tonifying drugs, blood-activating menstrual-regulating drugs, and heat-clearing and heat-cooling blood drugs, and most of them are classified as tonic drugs, blood-activating and removing blood stasis drugs, and heat-clearing drugs. (4) Medication clustering: 35 Chinese medicines with medication frequency ≥20% are divided into 11 categories, which are commonly used drug combinations for the clinical treatment of T2DM by Professor Xu Yunsheng. (5) Using the improved Apriori algorithm: the minimum confidence level of 0.5 is selected, data mining is conducted on all type 2 diabetes cases, and 21 prescriptions involving 10 Chinese medicines are unearthed, which are the basic prescriptions for the treatment of T2DM. Due to time and funding reasons, the number of cases included in this project is not ideal, resulting in biased results. It has not only discussed the use of drugs based on syndrome differentiation and symptomatic medication, but only discussed the rule of medication for diseases as a whole. In the follow-up research, it is necessary to further increase the number of cases collected and analyze the T2DM syndrome differentiation and symptomatic medication rule analysis to make the results more rigorous, systematic, and accurate.

## Figures and Tables

**Figure 1:** SAS data analysis software.

**Figure 2:** Gender distribution.

**Figure 3:** Age distribution.

**Figure 4:** Frequency distribution diagram of the four Qi of traditional Chinese medicine.

**Figure 5:** Frequency distribution diagram of five flavors of traditional Chinese medicine.

**Figure 6:** Frequency distribution diagram of ten kinds of Chinese medicine.

**Table 1:** Drug cluster analysis.

Class	ROC	RQN	1 − *R*^2^
1	0.62	0.16	0.45
2	0.36	0.06	0.67
3	0.90	0.18	0.12
4	0.74	0.16	0.31
5	0.71	0.23	0.38
6	0.40	0.04	0.62
7	0.94	0.13	0.06
8	0.57	0.07	0.46
9	0.59	0.33	0.61
10	1.00	0.16	0.00
11	0.47	0.10	0.59

## Data Availability

The datasets used and analyzed during this study are available from the corresponding author upon reasonable request.
